This article has been retracted.

# Identification of Prognostic LncRNAs Subtypes Predicts Prognosis and Immune Microenvironment for Glioma

**DOI:** 10.1155/2022/3709823

**Published:** 2022-10-07

**Authors:** Fei Chen, Xing Peng, Zhipeng Teng, Haibo Long, Haibo Wu

**Affiliations:** Department of Neurosurgery, Chongqing Traditional Chinese Medicine Hospital, Chongqing, China

## Abstract

Glioma is the most commonly occurring primary neuroepithelial neoplasm. Long noncoding RNAs (lncRNAs) are emerging as pivotal modulators of gene expression in the immune system and play critical roles in the growth, progression, and immune response of carcinomas. In this study, we performed univariate Cox regression analysis on survival data from TCGA and identified 20 prognostic lncRNAs. Moreover, we revealed that these prognosis-related lncRNAs (PRLnc) were dysregulated in glioma. Furthermore, we constructed a signature based on the expression levels of these prognosis-related lncRNAs based on 13 prognostic lncRNAs, including AGAP2-AS1, CYTOR, MIR155HG, LINC00634, HOTAIRM1, SNHG18, LINC01841, LINC01842, LINC01426, MIR9-3HG, TMEM220-AS1, LINC00641, LINC01270, and LINC01503. The Kaplan–Meier curves show that high-risk patients had a shorter survival time. Finally, the glioma samples were classified into 2 subgroups based on the median expression of prognosis-related lncRNAs in each sample. In summary, these findings suggest that PRLnc is associated with tumor-infiltrating immune cells in glioma and that subtype 2 patients may respond more positively to immunotherapy.

## 1. Introduction

Glioma is the most commonly occurring primary neuroepithelial neoplasm, mainly, occurring in the brain and arising in the glial tissue. The glioma family is consisting of ependymomas, astrocytomas (such as glioblastoma), oligodendrogliomas, mixed gliomas, and optic nerve, and brain stem gliomas, etc. [1]. The histology of these neoplasms varies greatly; from benign ependymal neoplasms to the most aggressive and fatal grade IV GBM [1, 2]. Although great advances have been made in the field of glioma therapies, comprising radiotherapy, chemotherapy, and targeted treatment, the treatment effect is still unsatisfactory, with a low success rate and 12–14 months survival period after treatment [3, 4]. Inaccurate disease progression prediction and unexpected treatment outcomes were probably due to complicated molecular mechanisms and inconsistent histopathological grading of glioma. At present, the standard treatment for patients with glioma is postoperative radiotherapy and adjuvant chemotherapy [5]. The need to uncover the molecules related to tumor development and to explore split-new methods for individualized treatment of patients with glioma is urgent [6].

Long noncoding RNAs (lncRNAs) exhibit important transcriptional activities, chromosome modification, and nuclear transport [7]. LncRNAs are widely distributed in various species and many kinds of human cells, with the features of stable structure, highly conservative, complex modulation, and tissue-specific expression [7]. There have been some studies showing that lncRNAs display as sponges to adsorb microRNAs (miRNAs) to modulate the expression of genes and exert an effect on regulating transcription and interfering with splicing mechanisms [8, 9]. More and more evidence showed that lncRNAs exhibited a pivotal role in tumor occurrence and metastasis [9, 10], including glioma. There were some studies demonstrating that lncRNAs played a role in glioma progression. For example, lncRNA HOXD-AS2 functioned as a promoter in glioma progression and was perhaps an outstanding target toward glioma's diagnosis and therapy [11]. LncRNA MT1JP mediated an inhibition of glioma cells growth, and metastasis via motivating the Akt signaling [12]. H19 imposed an effect on the immune infiltration level, thereby affecting glioma patients' prognosis [7]. Wang et al. reported that lncRNA LINC00473 might be expressed as a competing endogenous RNA (ceRNA) to decrease the level of miR-195-5p, followed by raising the expression of YAP1 and TEAD1, which were the downstream targets of miR-195-5p [13]. This finding sheds light on the working mechanisms of LINC00473, causing the progression of glioma [13]. LncRNA LINC00174 induced glioma glycolysis via modulating miR-152-3p/SLC2A1 [14]. Zhang et al. discovered that lncRNAs worked as epigenetic mediator and predictor in the proliferation, migration, invasion, angiogenesis and metastasis in cell line/animal model of glioma [15]. In summary, the studies listed herein make a compelling case for further investigation of lncRNAs in glioma. More promising lncRNAs associated with glioma need to be unearthed.

Herein, we carried out integrated bioinformatics to systematically investigate the association between lncRNA expression levels and glioma patients' clinical characteristics and the prognostic value of lncRNAs. We identified prognostic lncRNAs in glioma utilizing two public databases, including the CGGA and TCGA datasets. Furthermore, based on the expression of these lncRNAs, a predictive signature and two molecular subtypes were developed and established. Additionally, the distribution of tumor-infiltrating immune cells in prognostic lncRNA-based glioma subtypes was estimated. We hoped that this study would aid in identifying patients who might benefit from immunotherapy and hence increase glioma patient survival.

## 2. Methods and Materials

### 2.1. Expression Profiles and Sample Information

The RNA-seq data, as well as clinical features of glioma patients, were downloaded and analyzed from TCGA data to discover changes in gene expression. Age, tumor status, surgery status, and grade were all documented along with the clinical data. No further ethics committee approval was required due to all data were acquired from TCGA.

### 2.2. Establishment of Risk Signature and Statistical Analysis

We identified lncRNAs with prognostic potential using a univariate Cox regression model. The candidate lncRNAs that were substantially connected to survival were then filtered out using the LASSO model [16], resulting in a risk signature. The risk score was computed based on the levels of 13 different lncRNAs. The “survival” R program was used to plot the receiver operating characteristic (ROC) curve, and the Area under Curve (AUC) value was calculated to measure the predictability of the results. SPSS 25.0 (IBM Corp., Armonk, N.Y., USA) and R software were used for all image creation and data analysis in this investigation.

### 2.3. Functional Enrichment Analysis

Functional enrichment analysis was performed to assess the potential roles of DEGs in different prognostic lncRNAs related subtypes with the DAVID system [17]. Significantly enriched function annotations were defined with a 2-sided P value of less than 0.01.

### 2.4. Identification of Molecular Subtypes of Glioma

To cluster prognosis-related lncRNAs, researchers utilized ConsensusClusterPlus [18] V1.48.0. Using the median values of prognosis linked lncRNAs expression; the Z-score was utilized to classify the TCGA dataset.

### 2.5. Estimation of Tumor-Infiltrating Immune Cells

We have used CIBERSORT algorithms [19] to quantify the immune infiltration differences between subtype 1 and subtype 2 groups to study the association between prognosis-related lncRNAs and tumor-infiltrating immune cells. The StromalScore, ImmuneScore, and microenvironment score were then calculated in the subtype 1 and subtype 2 groups to evaluate the tumor microenvironment difference between the 2 groups using CIBERSORT algorithms. The Spearman's correlation test was performed to assess the correlations between PRLnc score and tumor-infiltrating immune cells, which were further, explored using the CIBERSORT algorithm. Moreover, the expression patterns of immune checkpoint genes in the two groups were then compared using the “ggpubr” package of R software [20].

## 3. Results

### 3.1. Identification of Prognosis Related lncRNAs in Glioma

Here, we determine the prognostic value of lncRNAs in glioma. We identified 20 prognosis-related lncRNAs (PRLnc) using a univariate Cox regression model, which was present as a forest map (Figure 1(a)). As can be seen from the figure, AGAP2-AS1, CYTOR, MIR155HG, MIR4435-2HG, HOTAIRM1, SNHG18, LINC01841, LINC01842, LINC01426, TMEM220-AS1, LINC01270, and LINC01503, LINC01273 were high-risk lncRNAs, which were significantly upregulated in glioma and positively correlated to the progression of glioma (Figure 1(b)). Whereas LINC00634, SLC25A21-AS1, MIR9-3HG, and LINC00641 were low-risk lncRNAs, which were suppressed in glioma and negatively correlated to the progression of glioma (Figure 1(b)).

### 3.2. Confirmation of the Correlation between PRLnc Expression and Outcome in Glioma Using CGGA Database

To confirm the correlation between prognosis-related lncRNA expression and overall survival (OS) time in glioma, we analyzed the CGGA database. As present in Figure 2, we showed the higher levels of AGAP2-AS1, CYTOR, HOTAIRM1, MIR155HG, and SNHG18 were correlated to shorter OS in patients with glioma, indicating these lncRNAs may serve as tumor promoting genes (Figures 2(a)–2(e)). However, higher expression levels of LINC00641, LINC00634, and SLC25A21-AS1 were correlated to longer OS in patients with Glioma, indicating these lncRNAs may serve as tumor suppressing genes (Figures 2(f)–2(h)).

### 3.3. Construction of an lncRNA Signature for Glioma

We next used LASSO regression analysis on these 20 lncRNAs to find the most promising candidates (Figure 3(a)). Finally, 13 lncRNAs were chosen as candidates for the lncRNA signature: AGAP2-AS1, CYTOR, MIR155HG, MIR4435-2HG, LINC00634, HOTAIRM1, SNHG18, LOC100506474, LINC01841, LINC01842, LINC01426, LINC01265, SLC25A21-AS1, LOC101928134, MIR9-3HG, TMEM220-AS1, LINC00641, LINC01270, LINC01503, and LINC01273 (Figure 3(a)).

The eight lncRNAs were combined to establish a risk score model for glioma patients, as follows: riskscore = (0.1434) ∗ AGAP2-AS1 + (0.1612) ∗ CYTOR + (4e − 04) ∗ MIR155HG + (−0.1641) ∗ LINC00634 + (0.0385) ∗ HOTAIRM1 + (0.0816) ∗ SNHG18 + (0.0141) ∗ LINC01841 + (0.0819) ∗ LINC01842 + (0.0016) ∗ LINC01426 + (−0.0282) ∗ MIR9-3HG + (0.0925) ∗ TMEM220-AS1 + (−0.1016) ∗ LINC00641 + (0.0768) ∗ LINC01270 + (0.0016) ∗ LINC01503 (Figure 3(a)). Individual risk scores were assigned to all patients based on the lncRNA signature.  Figure 3(b) depicts the correlation between the lncRNA expression and the risk score. We found high-score glioma patients have a shorter OS than low-score glioma patients (Figure 3(c)). We then performed time-dependent ROC curve analysis to determine the PRLnc signature in predicting the OS of glioma patients. The AUC was 0.88, 0.91, and 0.842 for 1-, 3-, and 5-years, respectively (Figure 3(d)). Our findings imply that the lncRNA signature established in this study is an effective biomarker of prognosis in glioma.

### 3.4. Analysis of PRLnc Expression to Identify 2 Subtypes of Glioma

Then, glioma were classified as 2 subtypes based on the expression of PRLnc expression using consensus clustering when *K* = 2 (Figures 4(a) and 4(b)). The samples were classified into 2 subgroups based on prognosis-related lncRNAs in each glioma sample (Figures 4(c) and 4(d)).  Figure 1 depicts PRLnc expression in the 2 subtypes of glioma (Figure 4(e)). Further examination of the correlations between the 2 subgroups and overall survival time revealed significant disparities in prognosis between the two subtypes. Those with subtype 1 glioma exhibited considerably shorter OS times than patients with subtype 2 glioma (Figure 4(f)).

### 3.5. Analysis of Differentially Expressed Genes between lncRNAs Related Subtypes in Glioma

We discovered DEGs between subtype 1 and subtype 2 glioma and created a volcano map to investigate the impact of prognosis-related lncRNA expression on malignancy. A total of 2398 DEGs were identified, with 1137 being induced and 1261 being suppressed (Figures 5(a) and 5(b)). The most significantly upregulated genes included CHI3L1, LTF, PDPN, MEOX2, TIMP1, IGFBP2, POSTN, EMP3, SAA1, METTL7B, RARRES2, FMOD, MOXD1, PLA2G2A, FABP5, NNMT, RBP1, and ANXA1. And the most significantly downregulated genes included SFRP2, SMOC1.

Figure 5 depicts the comparative values of the three datasets. The bioinformatics analysis showed upregulated DEGs were related to immune response, such as T cell activation, cellular response to IFN-*γ*, IFN-*γ*−mediated signaling pathway, neutrophil activation involved in immune response, neutrophil degranulation, and cell cycle, such as microtubule cytoskeleton organization, mitotic nuclear division, and mitotic sister chromatid segregation (Figure 5(c)). The bioinformatics analysis showed downregulated DEGs were related to axonogenesis, cognition, glutamate receptor signaling pathway, modulation of chemical synaptic transmission, neurotransmitter secretion, ion transmembrane transport, and membrane potential (Figure 5(d)).

### 3.6. Analysis of Tumor-Infiltrating Immune Cells Distribution in PRLnc Subtypes

We have used CIBERSORT algorithms to quantify the immune infiltration differences between subtype 1 and subtype 2 groups to study the association between prognosis-related lncRNAs and tumor-infiltrating immune cells.  Figure 6(a) depicts a heatmap of all significantly distinct immune responses. Comparative assessments of immune cell subpopulations indicated considerable disparities in immune cell infiltration levels between the subtype 1 and subtype 2 groups. We revealed the infiltrating levels of hematopoietic stem, endothelial cells, CD8+ naive T cells, common lymphoid progenitor, CD4+ Th2 T cell, macrophage, macrophage M1/2, monocyte, CD4+ memory T cells, CD4+ effector memory T cells, and CD8+ effector memory T cells were higher in subtype 1 than in subtype 2 groups. However, the infiltrating levels of NK cell, B cells plasma, CD4+ Th1T cells, myeloid dendritic cell activated, mast cell, T cells regulatory (Tregs), eosinophil, neutrophil, and T cell NK were higher in subtype 2 than in subtype 1 groups (Figure 6(a)).

StromalScore, ImmuneScore, and microenvironment score were then calculated in the subtype 1 and subtype 2 groups to evaluate the tumor microenvironment difference between 2 groups. The results showed that StromalScore, ImmuneScore, and microenvironment score were significantly higher in subtype 1 than in subtype 2 groups (Figures 6(b)–6(d)). Moreover, the correlations between PRLnc score and tumor-infiltrating immune cells were further explored, and the results showed that PRLnc score were significantly positively correlated to T cells CD8+ cells, neutrophil cells, macrophage cells, myeloid dendritic cells in glioma (Figure 6(e)).

The patterns of immune checkpoint genes in the two groups were then compared, and we observed several genes (CD274, CTLA4, HAVCR2, LAG3, PDCD1, PDCD1LG2, TIGIT, and SIGLEC15) were overexpressed in the subtype 1 group (Figure 6(f)). The TIDE algorithm was also utilized to determine whether PRlnc-related subtypes might predict immunotherapeutic benefit. Patients in the subtype 1 group showed considerably higher TIDE ratings than those in the subtype 2 group (Figure 6(g)), indicating that patients in the subtype 2 group might respond better to immunotherapy.

## 4. Discussion

Accompanied by the development of high throughput sequencing technology, studies towards the molecular basis of carcinoma have made progress, but the etiopathogenesis and biomarkers of glioma have not been completed [21, 22]. To ameliorate the curative effect and to clearly comprehend the pathogenesis of glioma, it is urgent to carry out more conclusive research to unearth the molecular biomarkers related to the initiation and progression of glioma and to identify potential therapeutic targets that are urgently needed. lncRNAs are a subset of RNA that is > 200 bps with limited or no protein coding ability. Increasing evidence shows that lncRNAs take part in glioma carcinogenesis, exhibiting as oncogenes or tumor suppressors. For instance, Ji et al. elaborated that lncRNA SChLAP1 stabilized ATN4 and stimulated NF-*κ*B signaling to induce the development of GBM by forming a complex with HNRNPL [23]. Another study demonstrated that LINC01116 mediated the facilitation of proliferation and neutrophil recruitment via modulating IL-1*β*, furnishing a novel understanding of lncRNAs-mediated glioma progression [24]. Besides, emerging evidence revealed that lncRNAs were abnormally expressed and their dysregulation exerted an effect on the occurrence and development of glioma. For example, Gong and Huang clarified that downregulated lncRNA maternally expressed gene 3 (MEG3) in glioma cells suppressed migration of glioma cells by modulating the miR-6088/SMARCB1 axis [25]. LncRNA LINC00909 was greatly raised in the tissues and cell lines of glioma, and it acted as a ceRNA to interact with miR-194 and thus up-regulate MUC1-C, further inducing cell proliferation and invasion of glioma [26]. Collectively, these findings demonstrate that lncRNAs play a crucial role in the occurrence and development of glioma and might act as a novel therapeutic target.

In our study, we identified 20 prognostic lncRNAs and revealed that these prognosis-related lncRNAs were dysregulated in glioma. It was suggested that AGAP2-AS1 overexpression was an unfavorable prognostic factor in many carcinomas, such as lung carcinoma and glioma [27–29]. In GBM, AGAP2-AS1 has been identified as an oncogenic gene that regulates GBM cell motility and invasion. Cytoskeleton regulator RNA (CYTOR), also known as LINC00152, is a new long intergenic noncoding RNA. As previously described, it was suggested that CYTOR was increased in gastric carcinoma [30], renal cell carcinoma (RCC) and gallbladder carcinoma tissues. As compared to paired noncancerous tissues, high expression of CYTOR exhibited a positive association with poor overall survival [31]. CYTOR was up-regulated in the tissues of hepatocellular carcinoma (HCC), with circulating CYTOR was also highly expressed in plasma specimens of HCC patients, and could be considered as a potential biomarker for HHC's diagnosis [32]. Zhenget al. elaborated that CYTOR was up-regulated in a variety of carcinoma types and is especially upregulated in GBM. The expression of SNHG18 exhibited a negative relation to the mutation of isocitrate dehydrogenase 1 (IDH1) [33]. Zheng et al. [33], revealed that SNHG18 promoted cell motility of glioma via disrupting nucleocytoplasmic transport of *α*-enolase. LINC01503 was greatly upregulated in the tissues and cells of glioma, and its overexpression exhibited a significant correlation with tumor size and WHO grade in patients with glioma. Mechanistic evaluation demonstrated that LINC01503 facilitated tumorigenesis and progression by activating Wnt/*β*-catenin signaling [34]. Recently, LINC01426 expression and function in human carcinomas have aroused great interest [35–37]. LINC01426 was upregulated in glioma, clear cell renal cell carcinoma, and lung adenocarcinoma, and the increased expression of LINC01426 was related to adverse clinicopathological characteristics. Functionally, LINC01426 played a pro-oncogenic role in these carcinomas, and it was reported to be implicated in regulating several neoplasms' biological phenotypes. Additionally, LINC01426 facilitated the progression of glioma by the PI3K/AKT signaling pathway and was an independent predictor of glioma patients' prognosis [37]. Little reports were shown towards these lncRNAs related to glioma, including LINC00634, LINC01842, LINC01265, LOC101928134, TMEM220-AS1, LINC00641, and LINC01270. However, there were other studies that revealed these lncRNAs displayed a relation to the process of other types of carcinomas. For instance, LINC01270 was shown to have a significant association with a worse outcome in breast cancer. This study further investigated LINC01270's functions and found that reduced LINC01270 dramatically inhibited cell viability, colony formation, and cell migration ability in triple-negative breast cancer (TNBC) cells. Li et al. suggested that inhibiting LINC01270 could give rise to the suppression of esophageal carcinoma (EC) progression via demethylation of GSTP1 [38]. Ablating LINC00634 resulted in a decrease in EC cell viability and an inducing in cell apoptosis levels [39]. In order to identify more accurate biomarkers for the prognosis of glioma, we aimed to construct a risk model based on the levels of these PRLnc. The 13 lncRNAs were combined to establish a molecular risk score model for patients with glioma. High-risk patients have a shorter life expectancy than their low-risk peers. We confirmed that the lncRNA signature established here is an effective predictor of overall survival in glioma patients. Based on AUC, the predictive performance of our risk score is better than in a previous study [40].

In 2016, the World Health Organization (WHO) incorporated molecular features into the classification of brain tumors for the first time to enable more accurate, “stratified” diagnoses, improve patient management, and more accurately estimate the likelihood of prognosis and treatment response. Based on their genetic profile, gliomas could be classified as IDH-mutant, 1p/19q-intact glioma. In this study, we identified molecular subtypes of glioma using prognosis-related lncRNAs expression in glioma samples. Finally, the glioma samples were classified into 2 subgroups based on the median expression of PRLncs in each sample. Those with subtype 1 glioma exhibited considerably shorter OS times than patients with subtype 2 glioma, indicating that the subtype 1 glioma patients may have a more aggressive cancer status.

Recently, research focusing on lncRNAs' function and acting mechanisms has been increasingly reported. LncRNAs play pivotal roles in the growth, progression, and immune system of carcinomas [41]. For instance, the lncRNA NeST was reported to have a relationship to T cell activation and was critical for the regulation of immune response [42]. The lncRNA NRON maintained T cells resting state via NFAT [43]. Carcinoma cell antigen presentation was downregulated by the oncogenic lncRNA LINK-A [44]. Li et al. found that the lncRNAs were related to immune cell infiltration and presented high tissue-specific expression [41]. Here, we identified several lncRNAs that are associated with immune pathways. We found that lncRNA-based subtype 1 and subtype 2 had distinct immune cell subpopulations. We found that the infiltrating levels of hematopoietic stem cells, endothelial cells, CD8+ naive T cells, common lymphoid progenitor, CD4+ Th2 T cells, macrophage, macrophage M1/2, monocyte, CD4+ memory T cells, CD4+ effector memory T cells, and CD8+ effector memory T cells were higher in the subtype 1 group than those in the subtype 2 groups. The TIDE algorithm analysis showed that patients in the subtype 1 group showed considerably higher TIDE ratings than those in the subtype 2 group, indicating that patients in the subtype 2 group might respond better to immunotherapy. Other noncoding RNAs might be valuable in the prediction of the prognosis of glioma [45–47].

In conclusion, we identified 20 PRLnc dysregulated in glioma. PRlnc is associated with tumor-infiltrating immune cells in glioma and that subtype 2 patients may respond more positively to immunotherapy. This study may help to identify glioma patients who will benefit from immunotherapy to improve their survival.

## Figures and Tables

**Figure 1:** Identification of prognosis related lncRNAs in Glioma. (a) A forest map showed 20 prognosis related lncRNAs (PRLnc) in glioma using a univariate Cox regression model. (b) The expression levels of PRLnc in glioma were evaluated.

**Figure 2:** Confirmation of the correlation between PRLnc expression and survival time in glioma using CGGA database. (a–h) The higher levels of AGAP2-AS1, CYTOR, HOTAIRM1, SNHG18, and MIR155HG, were correlated to shorter OS, However, higher expression levels of LINC00634, SLC25A21-AS1, and LINC00641 were correlated to longer OS in patients with glioma.

**Figure 3:** Construction of an lncRNA signature for glioma. (a) LASSO regression analysis on these 20 lncRNAs. (b) Figure 3(b) depicts the correlation between the lncRNAs expression and the risk score. (c) Kaplan–Meier analysis showed high-risk patients have a shorter OS than low-risk patients. (d) We then performed time-dependent ROC curve analysis to assess the ability of the PRLnc signature in predicting the OS of glioma patients.

**Figure 4:** Analysis of PRLnc expression to identify four subtypes of glioma. (a-b) Consensus clustering cumulative distribution function (CDF) and relative change in the area under the CDF curve (CDF Delta area) were analyzed. (c) The samples were classified into 2 subgroups based on prognosis-related lncRNAs in each glioma sample. (d) Principal component analysis (PCA) of 2 subgroups based on prognosis-related lncRNAs in each glioma sample. (e) The expression levels of PRLnc in 2 subgroups were presented. (f) Those with subtype 1 glioma exhibited considerably shorter OS times than patients with subtype 2 glioma.

**Figure 5:** Analysis of differentially expressed genes between lncRNAs related subtypes in glioma. (a-b) volcano map and heatmap showed DEGs between subtype 1 and subtype 2 glioma samples. (c-d) GO analysis of upregulated and downregulated DEGs.

**Figure 6:** Comparison of PRLnc subtypes and existing immune molecular subtypes. (a) Heatmap was used to depicts of all significantly distinct immune infiltration levels by using CIBERSORT algorithms. (b–d) microenvironment score, StromalScore, and ImmuneScore, were then, examined in the two groups. (e) The correlations between PRLnc score and tumor-infiltrating immune cells were calculated. (f) The expression patterns of immune checkpoint genes in the two groups were then compared. (g) The TIDE algorithm was also utilized to determine whether PRlnc related subtypes might predict immunotherapeutic benefit.

## Data Availability

The data used to support the findings of this study are available from the corresponding author upon request.
